# Smart Bracelet System for Temperature Monitoring and Movement Tracking Analysis

**DOI:** 10.1155/2021/8347261

**Published:** 2021-07-20

**Authors:** Bin Fang, Fuchun Sun, Zhou Quan, Huaping Liu, Jianhua Shan

**Affiliations:** ^1^Beijing National Research Center for Information Science and Technology, Department of Computer Science and Technology, Tsinghua University, Beijing, China; ^2^Anhui Province Key Laboratory of Special Heavy Load Robots, Anhui University of Technology, Ma'anshan, China

## Abstract

In several epidemic diseases, one of the main symptoms exhibited by people is abnormal body temperature. Therefore, monitoring body temperature is crucial for preventing the spread of infectious diseases and facilitating timely responses. This study presents a wearable bracelet that can be used as a temperature monitoring and trajectory analysis system. The temperature sensor in the bracelet can effectively monitor the body temperature of the wearer in the target scene, and the data transmission between the bracelet and the data collector can effectively detect the movement range and trajectory of the wearer. Through these, the whole set can also detect the direct and indirect contact of the wearer in any period of time, which is very helpful for the prevention and control of infectious diseases and the isolation of potentially infected persons.

## 1. Introduction

COVID-19 is a new infectious disease that has caused enormous economic losses around the world because of its long incubation period and strong infection capabilities. Effectively isolating the virus and ensuring the safety of human lives have become a top priority. For such extremely infectious diseases, screening potential infectors according to their symptoms would be of great significance for the prevention and control of epidemics.

Similar to COVID-19, a main symptom of many infectious diseases, such as influenza, SARS, MERS, plague, and cholera, is fever [1], and this study showed that half of the COVID-19 patients had a body temperature above 37°C on admission and 78.5% of the study population had a body temperature above 37°C during the onset of the disease [2]. Therefore, a system for monitoring body temperatures of individuals would be very useful in the prevention and control of infectious diseases.

Many researchers have proposed various methods for detecting human body temperatures. Al-Hossain et al. proposed a contactless syndromic surveillance platform for influenza-like illnesses in hospital waiting areas called FluSense [3]. This system uses thermal imaging technology to detect body temperatures of individuals in hospitals. Fajrin et al. proposed a telemedicine system that collects body temperature data using DS18B20 sensors and then processes the data using an Atmega328 microcontroller before sending the results to mobile phones via Bluetooth [4]. Yang and Zheng proposed the use of wireless low-power thermal sensors for basal body temperature detection based on frequency-modulated telemetry devices. Their devices adopt a temperature compensation mechanism and achieve good results for the measurement of human body temperature [5]. Although these methods have been applied in various scenarios, they still suffer from some significant limitations. For example, Liu et al. demonstrated the limitations of temperature detection methods that use forehead surface temperature [6].

Temperature monitoring in communities and schools around the world is largely performed using point temperature measurement solutions, such as temperature guns, infrared thermometers, and thermal imagers. However, such methods have numerous problems, including crowding, tedious temperature measurement, and statistical limitations; this implies that there are still significant blind spots from the perspective of epidemic control.

With the development of sensor and communication technologies in recent years, wearable devices have begun to play an important role in our daily lives. Many researchers have used data collected by various wearable sensors to perform different types of research. Gu et al. used sensor data and Wi-Fi technology to continuously monitor sleep patterns [7]. Vhaduri et al. proposed a method that uses data collected by smartphones and sensors to opportunistically fill gaps in user location traces [8].

As one of the most widely used wearable devices, smart bracelets have become an important part of the daily life of many people. Such bracelets can be used to monitor sleep patterns and heart rates and also to calculate running speeds [9]. Many researchers have performed studies based on the data collected by smart bracelets. Nguyen et al. performed daily wrist activity recognition using smart bracelet data [10]. Heart rate data collected from smart bracelets have been used for emotional analysis [11] and health status monitoring [12]. Smart bracelets also play an important role in gait analysis of the elderly [13] and urination analysis of patients with certain diseases [14].

In this study, we propose a community temperature monitoring system using smart bracelets which can accurately measure body temperatures of wearers. This system requires several data collectors to be installed on campuses or communities, which can serve as base stations to locate wearers. Temperature data of wearers can be rapidly collected, and their locations can be determined by regular reporting of collected data. Using this system, monitoring personnel can rapidly screen people with infectious diseases so that efficient measures for disease prevention and control can be taken. This system can collect large amounts of body temperature and location data every day and only requires users to wear bracelets; thus, it can avoid the aggregation problem while detecting body temperature, which is of great significance for disease prevention and control. Other methods can only screen direct contacts, whereas our system can effectively screen all direct and indirect contacts of potentially infected individuals.

## 2. Related Work

COVID-19 is still rapidly spreading worldwide. To control this epidemic effectively, many research institutions and companies have developed their own systems for monitoring human body temperature and tracking human movement.

For example, Singapore launched a system called TraceTogether [15]. The working principle of TraceTogether is to exchange short-range Bluetooth signals between mobile phones (devices are required to always have their Bluetooth functions activated for this) to detect other users of TraceTogether within short distances. These close contact records are then stored on each user's mobile phone; collected data are encrypted. The data are not uploaded through a network; only if users are diagnosed with an infection will the government ask them to provide data collected on their phone so they can track other individuals who have been in close contact with them. The Ministry of Health can then notify those individuals using TraceTogether so that they can monitor their own health and check whether they are exhibiting any symptoms of the infection; this allows them to receive proper guidance and care.

Apple and several US federal agencies have launched an app and a website, as a screening tool, called Apple COVID-19 [16]. This app is mainly used to provide guidance to users regarding COVID-19 by the US Center for Disease Control. By using this app, users can understand the risks within their scope of influence so that they can respond in a timely manner. Additionally, general COVID-19 information and proper protection measures are also available on this app.

In June 2020, an app called Corona-Warn, supported by the German federal government and German companies SAP and Telekom, was launched [17]. This application uses Bluetooth technology to send signals within a few meters. Users can learn if there are infected individuals nearby through push notifications. For example, if person A is infected, their device sends a warning message to all nearby mobile phones with this app installed through push notifications, thereby warning users of this app.

Although these systems and apps can be very useful for epidemic prevention and control, they still pose several limitations. For example, such systems rely entirely on mobile phones, which implies that individuals without smartphones cannot be factored into the analysis. Additionally, all the systems described above use Bluetooth technology, which requires users to keep their Bluetooth feature turned on, which can be a threat to personal privacy. Due to these issues, many users have concerns regarding personal privacy protection when using these systems.

There are many different control methods available for managing temperature monitoring systems.  Figure 1 summarizes the issues of various methods. Our system was developed as an attempt to resolve these shortcomings.

## 3. Proposed System

The proposed system mainly consists of wearable smart bracelets and data collectors. Data collectors are installed at fixed locations. The proposed system can be used in government agencies, schools, and aggregated office spaces.

The proposed workflow for a detection and tracking model is presented in Figure 2. First, body temperatures of smart bracelet wearers are measured. Next, data collectors collect wirelessly transmitted data from the smart bracelets. Finally, data are uploaded to a cloud platform, on which abnormal temperatures and activity ranges are analyzed. This system only uses data collected by the smart bracelets to avoid private data leakage associated with mobile phones. Each bracelet has a unique ID and a corresponding wearer ID. The list of IDs can only be obtained by a system administrator. Additionally, the application scope of the proposed system is limited to designated office or community spaces to avoid leakage of user location information. Therefore, even if a smart bracelet is lost, personal information of the original wearer cannot be obtained.

As shown in Figure 3, our smart bracelet consists of nine main modules: a liquid crystal display (LCD) module, power management module, charging module, 2.4 G communication module, main control system module, temperature measurement module, data storage module, touch management module, and clock management module. These modules can provide not only the temperature measurement functionality but also basic smart bracelet functions to wearers.

Using radio frequency (RF) technology, a smart bracelet can transmit data to data collection and processing devices. RF technology is a noncontact automatic identification technology. Its basic principle is to use the transmission characteristics of RF signals and electromagnetic coupling for automatic identification of target objects. Therefore, when a smart bracelet enters the wireless connection range of a data processing device, it can connect to the data processing device wirelessly and automatically. Additionally, a data processing device can identify smart bracelets of multiple wearers simultaneously. In the application scenario considered in this study, the bracelets are connected via RF technology to data collection devices. Bluetooth can also be used for data transmission in other application scenarios.

When a smart bracelet is worn correctly, the temperature measurement module will be in contact with the wearer's body, allowing it to obtain his/her body temperature. Then, the acquired data will be sent to the main control chip (main control system module), which transmits the data via the wireless transmission module. Finally, the data are transferred to a data collector for further analysis.

Each smart bracelet also has a touch screen (LCD module), which shows the users their body temperature data in real time; furthermore, users can interact with the system through the touch management module. The power system consists of power management and charging modules for optimal power consumption. In addition, the sustainable working time of smart bracelet is one week. The data storage module is used to record daily temperature data and other routine data from users. The clock management module is used to provide users with basic time information.

For better detection and acquisition, we imposed some regulations on smart bracelet wearing:

1. It is suggested to wear it on the inside of wrist to improve the measurement accuracy.
2. Please avoid testing within 30 minutes after exercise or bathing.
3. Please avoid wearing too tight or too loose, so as not to affect the test results.
4. This product cannot replace the doctor's diagnosis, only for screening. If there is any abnormality, please see a doctor in time.

### 3.1. Data Collector

In our system, data collectors are connected to smart bracelets via RF technology, which can realize readout operations in the smart bracelets. In the application scenario considered in this study, the wireless connection range is limited to approximately 15 m to ensure data acquisition stability.  Figure 4 presents the components of our data collectors. A data collector contains receiving and transmitting antennas outside the shell. These antennas are used to read signals from the smart bracelets and send results of temperature data analysis to the smart bracelets. As shown in Figure 5, a data collector can also be used to determine the number of users in a particular area. Additionally, according to differences in signal strengths, the relative positions of the users and data collectors can be roughly estimated.

A data collector consists of a temperature sensor that detects external environmental temperature; this is used to process temperature data collected by smart bracelets. The temperature sensor and data processing device are connected to the main component through a circuit and a temperature detector component extends outward. The temperature sensing component is exposed to the external environment so that it can transmit the detected ambient temperature to the data processing device. The temperature sensor is a thermistor; its resistance value changes with changes in temperature. When the temperature increases, its internal resistance decreases; thus, the detected current will increase. By detecting the magnitude of the current, the temperature of the surrounding environment can be determined. The data processing device compiles the ambient temperature into an electronic signal that can be transmitted through the Internet of Things card circuit. The data uploaded by the data processing device consists of the compiled ambient temperature and body temperature data, which are transmitted to the background management equipment. Next, temperature compensation calculations are performed in the background management equipment, allowing background management personnel to determine the temperature information of users within the system detection range.

For better detection and acquisition, we imposed some regulations on data collector locations:

1. A data collector should be placed in an open and cool location to facilitate accurate collection of ambient temperature data.
2. The antenna of a data collector should be as far from walls and metal shell as possible to avoid negatively affecting signal receiving distance.
3. The usage environment of the data collector should be such that mobile network signals of appropriate frequency bands are available for effective communications.
4. The number of data collectors receiving data from smart bracelets simultaneously is limited and should not exceed 150. Additionally, the receiving distance should not be greater than 15 m.
5. Data collectors should be placed in individual rooms to avoid partitioning transmissions as much as possible.

To achieve effective monitoring of human body temperature and save system resources, we set different upload intervals for data collectors in different locations. For example, at a school gate, considering the mobility of the target crowds, the upload interval was 60 s. In classrooms and dormitories, the upload interval was 480 s.

### 3.2. Temperature Estimation

Temperature measurements on the wrist fluctuate significantly with external temperature. Therefore, a temperature compensation formula was defined as follows:

(1) $$\begin{array}{c} T_{B}=f\left(T_{E},T_{M}\right), \end{array}$$

where *T*_*B*_ is the body temperature, *T*_*E*_ is the environmental temperature, *T*_*M*_ is the original measured temperature, and *f* is the mapping function.

In daily temperature measurements, a variety of factors may result in temperature measurement errors. To achieve suitable temperature measurement performance, we performed various operations. First, we collected a portion of the original smart bracelet temperature measurement data, environmental temperature data, and mercury thermometer temperature measurement data. We then calculated the means and variances of the wrist temperature data (measured by smart bracelets) and environmental temperature data; we used the data to generate body temperature data with a normal distribution. Finally, we considered the temperatures measured by a mercury thermometer as accurate values and used the generated data to fit the accurate values using the least-squares method. Based on the randomness and noise in the generated data, the generalization ability of the fitting equation was improved to a certain extent using the generated normal data to fit actual body temperature measurements.

(2) $$\begin{array}{c} T_{E}=g\left(T_{E}^{\prime }\right),\\ T_{M}=g\left(T_{M}^{\prime }\right),\\ T_{B}=a\times T_{E}+b\times T_{M}, \end{array}$$

where *g* is the generation function for the normal distribution; *T*′_*E*_ and *T*′_*M*_ are the original temperature data; and *a* and *b* are the fitting coefficients, which are equal to 0.32 and 0.82, respectively (Algorithm 1).

In addition, we verify the whole system in extreme weather. When the temperature is higher than 50°C and the sunlight is too strong, the temperature rise of the hardware surface will have a negative impact on the measurement accuracy.

### 3.3. Contact Tracing System

The bracelet can receive the wireless connection request from the data collector (base station) within the connection range. After the verification of the wireless connection request, the bracelet returns a consent connection response to trigger the base station to establish a wireless connection with the bracelet itself. Through wireless connection, the detection data is sent to the base station to make the base station acquire the detection data, and send the detection data, the connection information between the base station and itself, and the disconnection information to the server, thereby triggering the server to obtain its own activity information at the predetermined address. Among them, the detection data includes the detection temperature, detection time, and its own unique identification; the connection information includes the starting connection time and the unique identification; the disconnection information includes the connection disconnection time and the unique identification. Through these ways, the system can track the crowd activities and find the close contacts quickly and accurately.

### 3.4. Data Confidentiality

For the body temperature data and other information collected from wearers, we constructed a data protection system that ensures that only authorized personnel can access personal data, which protects user privacy:

1. Management level: to ensure that the business model of the proposed system functions properly, a confidentiality management organization is established; it consists of full-time personnel to control confidentiality management tools. The confidentiality system and tools are integrated into all levels of the business process to reduce the number of unnecessary links that could lead to leakage. If a leak occurs, it can be located rapidly by considering the responsible party as the target point and the corresponding business process as the line to the target point.
2. Hardware level: the proposed system is capable of monitoring, communicating, office automation, safety detection in electromagnetic environments, and securing the confidentiality of computer networks using human, physical, and technical preventive measures.
3. Technical level: an asymmetric encryption algorithm is used to encrypt data, and cryptography is used to protect data security. Daily maintenance of the system strictly follows the process operation schedule to ensure that information is not leaked to/tampered with by unauthorized users or entities during the processes of storage, usage, and transmission. Additionally, the proposed system can prevent authorized users from tampering with information or the system itself, which ensures the security of data.

## 4. Analysis and Results

By using the proposed system, we can collect large amounts of body temperature data and other information daily. On average, hundreds of thousands of pieces of data are generated every day. This volume of data is significant for mining potential relationships using big data tools.

In this study, we consider a system deployed in a primary school as an example and all participants were about 2000. Each smart bracelet corresponds to a student, teacher, or school worker and each data collector corresponds to a location. We have shown locations and corresponding IDs in Table 1 for better clarity.

As shown in Figure 6, we consider data from June 1 to June 27. Significant reduction in the amount of uploaded smart bracelet data is seen on weekends and vocational days (Chinese traditional festival called the Dragon Boat Festival); this corresponds to typically observed trend on weekends and other holidays.

### 4.1. Temperature Analysis

As shown in Figure 7, the temperature data calculated by our system based on environmental temperature and body surface temperature data are closer to the values measured with a mercury thermometer than those obtained by other methods; this implies that our system has relatively higher accuracy of body temperature measurement.

This work proposed that changes in oral/rectal and axillary temperatures correlated significantly (*p* < 0.0001) [21]. Considering that oral/rectal temperature measurement may be more likely to cause virus infection and in order to demonstrate the effectiveness of our measurement method, we consider armpit temperature values measured by a mercury thermometer as reference values and compare the values obtained by our method to those obtained by other methods. We obtain the body temperature of these methods by taking three different temperature measurement methods for the same patient in the hospital. In addition, there are some ways to make sure the data reliability. (1) The bracelets are worn all the time when patients are in hospital. (2) When the hospital uses its own equipment to measure the user's temperature, use the bracelet host with the same number as the bracelet to measure the user's armpit temperature, and make a record. (3) The number of measurements should be as many as possible, with an average of no less than 5 times a day.

As shown in Table 2, the mean absolute error (MAE) and mean-squared error (MSE) for our measurement method are smaller than those of some other measurement methods.

Because the example system is deployed in a school, only few teachers or staff will upload data during weekends. For detailed analysis, we considered a sample of smart bracelet data.  Figure 8 presents the curves of body temperature and surface temperature for a particular user during a working day. The proposed system can be used to monitor a user's temperature using these data. When a user's body temperature is abnormal, the system will query the smart bracelet number and locate the user based on the data collector that uploaded the corresponding data.

### 4.2. Crowd Distribution Analysis

By using the proposed system, we can determine the number of people in a certain classroom or entrance.  Figure 9 presents a schematic of the system statistics for the number of people in a room. Because the collection range of each data collector is one room or entrance, the number of people in a particular room can be determined according to the number of bracelets' uploading data to the corresponding data collector. Using the data shown in the figure, the number of people in a specific place can be monitored and an alarm can be initiated when that number exceeds a predefined threshold; this can effectively reduce the potential risk of infection caused by crowds.

### 4.3. Contact Tracing Analysis

Many methods use Bluetooth connections for contact tracing. Specifically, when a user is within the range of another user's Bluetooth device, a record is generated. However, such methods require users to keep their Bluetooth functions turned on at all times, which increases the risk of a leak of personal information.

In our system, users can be traced to specific locations. Because data collectors only collect smart bracelet data within a small range, users who have been in contact with other infected individuals can be identified.  Figure 10 presents the workflow of the movement and contact tracing system.

First, we determine which data collectors were used by the target smart bracelet to upload data. We can then query the locations of these data collectors to determine the movement of the user. Finally, by querying the IDs of the bracelets that a base station has connected to within a certain time range and querying the corresponding personnel information, we can identify anyone who has had direct/indirect contact with an infected user.

For a more detailed explanation, we consider bracelet No. 00010221 as an example. On June 9, this smart bracelet uploaded its data to the following data collectors: No. 1537, No. 1487, No. 1574, No. 1456, No. 1365, No. 1540, No. 1564, and No. 1405. From Table 1, we can determine that the wearer of this bracelet visited the following locations in order: class 2, grade 2; dean's office; science classroom; class 1, grade 3; class 2, grade 6; teacher's office; class 2, grade 4; and class 1, grade 2. If we want to identify this user's direct or indirect contacts, we only need to query the IDs of the bracelets that uploaded data to these data collectors on the same day.

In Figure 11, each line represents a user's tracking record. Assuming that the red line represents an infected patient, direct or indirect contacts can be identified by determining the intersection points of the tracking records of this user and other users. If a connection between two users does not exist, it means that they did not come in contact with each other.

## 5. Conclusion

In this study, we presented a group temperature measurement and contact tracing system using wearable smart bracelets. Compared to other methods/systems, our proposed system has lower deployment cost, is easier to operate, and can better protect user privacy. Compared to some systems that rely on Bluetooth technology, which can only screen individuals who have had direct contact with a person, our system can screen all potential contacts more comprehensively. The proposed system can collect user temperature data and location data in real time through smart bracelets. Because the bracelets do not store personal information, the proposed system avoids leakage of personal information in case the bracelet is lost. We used temperature sensors in the bracelets to measure relative body temperature and temperature sensors in data collectors to measure relative environmental temperature. We then combined these measurements to evaluate true body temperature, which significantly improves the measurement accuracy. This system also has some problems to be solved; for example, the disinfection of the surface of the bracelet may increase the workload, and it is only suitable for small-scale community use at present. The future research direction is to expand the application scope of the whole system and improve the universality of the whole system for different application scenarios.

## Figures and Tables

**Figure 1:** Research status analysis [15–20].

**Figure 2:** System description: (a) components of the proposed system; (b) control process for abnormal body temperature.

**Figure 3:** Components of the proposed smart bracelet.

**Figure 4:** Components of a data collector.

**Figure 5:** Room crowd statistics system.

**Figure 6:** Smart bracelet data uploaded over four weeks (June 1 to June 27).

**Figure 7:** Body temperature values measured by different methods.

**Figure 8:** Body temperature curve of a wearer during a working day.

**Figure 9:** Crowd statistics system.

**Figure 10:** Movement and contact tracing system.

**Figure 11:** Contact tracing example.

**Algorithm 1:** Pseudocode.

**Table 1:** Location and corresponding IDs.

Place	Dean's office	Teachers' office	Science classroom	Canteen	Reception room	Class 1, grade 1
Corresponding ID	1487	1540	1574	1398	1363	1538
Place	Class 2, grade 1	Class 1, grade 2	Class 2, grade 2	Class 1, grade 3	Class 2, grade 3	Class 1, grade 4
Corresponding ID	1534	1405	1537	1456	1576	1558
Place	Class 2, grade 4	Class 1, grade 5	Class 2, grade 5	Class 1, grade 6	Class 2, grade 6	
Corresponding ID	1564	1543	1514	1479	1365	

**Table 2:** Temperature measurement using different methods.

Measurement methods	MAE (°C)	MSE ((°C)^2^)
Estimated temperature	**0.41**	**0.30**
Forehead temperature device	3.18	11.86

## Data Availability

For the body temperature data and other information collected from wearers, the authors constructed a data protection system that ensures that only authorized personnel can access personal data, which protects user privacy.

## Appendix

In addition to COVID-19, this system has a certain role in the prevention of other infectious diseases that can cause abnormal body temperature, like plague, cholera, SARS, MERS, poliomyelitis, and some other infectious diseases.
